# Improved Faster R-CNN Based Surface Defect Detection Algorithm for Plates

**DOI:** 10.1155/2022/3248722

**Published:** 2022-05-17

**Authors:** Baizhan Xia, Hao Luo, Shiguang Shi

**Affiliations:** School of Computer, Zhongshan Institute, University of Electronic Science and Technology of China, Zhongshan 528402, China

## Abstract

Defect recognition plays an important part of panel inspection, and most of the current manual inspection methods are used, but the recognition efficiency and recognition accuracy are low. The Fast-Convolutional Neural Network (Faster R-CNN) algorithm is improved, and a surface defect detection algorithm based on the improved Faster R-CNN is proposed. Firstly, the algorithm improves the bilateral filtering algorithm to smooth the image texture background. Subsequently, a feature pyramid network with a shape-variable convolutional ResNet50 network can be applied to acquire defect semantic feature maps to improve the network's ability to express the features of multiscale defects while solving the difficulty problem of many types of defects and variable shapes. To obtain more accurate defect localization information, the algorithm in this paper uses the Region of Interest Align (ROI Align) algorithm instead of the crude Region of Interest Pooling (ROI Pooling) algorithm. Then, an improved attention region recommendation network is used to improve the focus of the model on plate defects and suppress the features of complex background. Finally, a K-means algorithm is added to cluster the defect data to derive anchor frames that are better adapted to the plate defects. In this paper, a dataset containing 3216 images of surface defects of plate metal is made by acquiring surface defect images from the production site of the plate metal factory, which mainly include various defect types. This dataset is used to train and test the algorithm model of this paper, and the results of detection accuracy and detection speed are compared with those of other algorithms, which prove that the algorithm of this paper can achieve real-time detection of plate defects with high detection accuracy.

## 1. Introduction

At present, China's home furnishing industry market is booming, and the 2020 annual output value of China's home furnishing industry is expected to reach 1 trillion yuan. The main driving force is that people pay more attention to the overall layout of housing space, design involvement, brand connotation, and health and environmental protection factors. Customized home furnishing is becoming more and more popular among consumers, so custom furniture is one of the most rapidly developing components of the home furnishing industry [1–3]. Despite the impact of domestic real estate regulation in recent years, custom furniture still maintains an annual growth rate of more than 20% and is expected to reach a market size of 2500 billion yuan by 2022. Under the traction of the strong demand, the order volume of manufacturing enterprises such as major raw material plate manufacturing enterprises and custom home furnishing enterprises continues to climb.

To meet the growing demand, much automated equipment is introduced in the panel production chain. At the raw material end, medium density man-made panels, high density man-made panels, and solid wood particle boards are commonly used as the main materials [4]. Inevitably, pits, bumps, oil spots, water spots, glue spots, chipped edges, bulging, and other problems are introduced in the processing process, which will directly affect the downstream surface lamination process. At the manufacturing end of the finished product, scratches, scrapes, knocks, chipped edges, dents, bulges, etc. will inevitably occur before the factory is installed by the end customer. The surface quality of man-made board directly affects the manufacturing quality of subsequent products. However, during the production process, some defects will inevitably arise. These defects can seriously affect the product quality and cause economic losses to the enterprise [5]. At present, most of the plate defect detection links use manual detection methods, while the continuous press production line of man-made board runs at high speed, the circulation of the plate is large, the manual detection work is intensive, easy to produce errors and omissions, and the detection rate is low. Therefore, there is an urgent need to provide a set of inspection methods to meet the real-time and high-precision requirements for detection of defects on the surface of man-made boards [6–8].

Machine vision is widely used for product surface defect detection due to its advantages of fast recognition and high accuracy [9]. Based on the machine vision artificial board defect detection system, the image is firstly acquired, and feature values are obtained. Then, the classifier is used to identify the defects based on the feature values. Finally, the defects are graded by their type and size [10]. The result of defect recognition directly affects the judgment of the board appearance quality. The continuous press production line has a speed of 1.5 m/s with intervals less than 0.4 m and a board area of 2.4 m × 4.8 m, which requires a high real-time performance and a judgment within 3 s. Therefore, a fast and accurate algorithm is needed for online detection and identification of defects in man-made boards.

Several detection methods based on classical visual data are available. In the literature [11], a pruned decision tree-based method for artificial board surface defect recognition was proposed. The method obtains the shape and texture features of defects as input by preprocessing and segmenting the existing artificial board defect images. The generated CART tree is pruned using a cost complexity algorithm, and finally the artificial board defects are recognized. In the literature [12], a wood defect recognition method with near infrared (NIR) spectroscopy and inverse neural network was proposed. In the literature [13], a method of classifying board defects by local binary mode and binary differential excitation mode was proposed. The method performs feature extraction by local binary differential excitation mode and uses a two-dimensional histogram for defect identification. There are also artificial board defect recognition methods based on region screening segmentation and random forest, artificial board surface defect detection image adaptive fast threshold segmentation algorithm, and artificial board surface image defect extraction method based on grayscale cogeneration matrix and hierarchical clustering. All of these methods require manual selection of certain key parameters or production features of the artificial board surface and have the disadvantages of low generalization ability and shallow feature level [14].

Deep learning [15], especially convolutional neural networks, with the advantages of deep feature hierarchy, high detection accuracy, and good robustness, has been gradually applied to defect detection in various fields [16]. Deep learning-based defect detection models fall into two main categories. One is regression-based methods, such as the SSD model. Literature [17] improved the VGG network part of the SSD model by replacing the VGG network using a deep residual network. The improved SSD model achieved an average detection accuracy of more than 89% for defects in fir and pine wood. Literature [18] used the DenseNet network to combine the improved SSD model and combined migration learning with the improved SSD model to achieve defect detection in wood with high accuracy. The other is region suggestion-based methods such as R-CNN model and Fast R-CNN model [19, 20]. Literature [21] designed a multichannel modal region convolutional neural network (Mask R-CNN) approach for wood detection, which can achieve high detection accuracy. Literature [22] combined adversarial generative networks with Mask R-CNN to achieve the recognition of defects such as dead and live knots in wood. Literature [23] applied the Faster R-CNN model to wood panel defect detection for the first time. The algorithm also uses multiple neural network models for migration learning to improve the performance of wood panel defect detection.

Based on the existing wood panel defect detection methods, we propose a new algorithm for panel surface defect detection. The algorithm uses the modules of pyramid network, attention region recommendation network, and region of interest calibration to improve the Faster R-CNN model, which makes the model have high detection accuracy for the panel defects in complex background.

Section 2 of the article is an introduction to man-made plates and defect categories.  Section 3 is an introduction to image preprocessing.  Section 4 is a specific introduction to the algorithm of this paper.  Section 5 is the algorithm experiment and analysis.  Section 6 is the conclusion.

## 2. Man-Made Panels and Defect Categories

In home customization, there are common panels including raw material panels, veneer panels, and finished panels. The following challenges exist in the identification of surface defects of these boards: first, there are many kinds of surfaces, and it is expected that there are as many as 5 kinds or more.  Figure 1 shows the schematic diagram of MDF/HDF raw material panels, particle board raw material panels, and veneer panels, respectively.

Second, the surface of the texture of many kinds of textures and complex textures are problems to be solved. Take the veneer panel as an example, usually a custom home furnishing enterprise produces as many as 40 kinds of panels, whose texture has different shades of color, shade, and shape, which brings great difficulties to the identification of its surface defects.

Third, there are many kinds of surface defects, including corner damage defects, edge damage defects, glue spots, oil spots, black spots, water spots, coarse fibers/shavings, cracks, coarse sand/sand leakage, slab edge sanding defects, sanding indentation, sand marks, pad marks, trembling marks, holes, pits, bulging, delamination, rough areas, pockmarks, trachoma, gaps, yin and yang, debris, and more than 20 kinds of defects. These defects are different in the performance of raw material panels and veneer panels. In addition to the difference in background material, even the same bulge is very different for the raw material board and the finished board at the image end.

Fourth, there is a certain openness in the types and manifestation characteristics of defects. With the plate processing and manufacturing work, the front-end manufacturing equipment and processes may bring new defect characteristics.

## 3. Image Preprocessing

In this paper, image preprocessing consists of two parts: texture background smoothing and data enhancement. Texture background smoothing is a texture smoothing algorithm that blurs the wood panel texture background to a certain degree while maintaining structural edge details to reduce the impact of complex and variable texture background on scratch defect recognition.

The wood panel surface has a complex and variable texture background, and the panel defects account for a small proportion of the whole image, both of which can affect the defect detection effect. Therefore, an appropriate texture smoothing algorithm is required during image preprocessing to blur the texture background to some extent while maintaining the details of the structure edges. This can increase the accuracy and robustness for detecting defects under different texture backgrounds.

Currently, texture smoothing is usually done using filtering methods, which are mainly classified as Gaussian filtering, bilateral filtering, and global optimization filtering algorithms. Gaussian filtering is better for texture background smoothing but leads to blurring of structure edge details, which is not good for defect feature retention. Global optimization filtering is required in the process of texture smoothing to ensure that the difference between the image after texture smoothing and the original image is minimized. Global optimization filtering can achieve strong gradient texture smoothing, with the disadvantage that it cannot smooth scale varying textures.

Bilateral filtering algorithm excels in the field of texture smoothing. Bilateral filtering is based on Gaussian filtering, considering both the gray value around the pixel point and the position relationship between the pixel points, and the pixel gray value calculation can be expressed as

(1) $$\begin{array}{c} m=\exp\left[-\frac{{\left(x-z\right)}^{2}+{\left(y-l\right)}^{2}}{2\sigma_{d}^{2}}-\frac{{\left\|X\left(x,y\right)-X\left(z,l\right)\right\|}^{2}}{2\sigma_{r}^{2}}\right],\\ X_{D}\left(x,y\right)=\frac{\sum_{z,l}X\left(z,l\right)m}{\sum_{z,l^{m}}}. \end{array}$$

where *x*, *y*, *z*, *l* are the pixel location coordinates. *X*(*x*, *y*) is the grayscale value of the (*x*, *y*) pixel point. *σ*_*d*_ is the smoothed weight value associated with the spatial location. *σ*_*r*_ is the smoothed weight value associated with the pixel. *X*_*D*_(*x*, *y*) is the grayscale value of the pixel point after smoothing.

After testing, it was found that the defects also became blurred after the bilateral filtering algorithm for the wood panel images. The reason is that the defect features are too fine, and the pixel gray value is easily blurred out by the surrounding pixel gray value. Therefore, the concept of pixel edge length is proposed and applied to the bilateral filtering algorithm in this paper. The improved algorithm considers the edge detail length relationship between pixel points in the weight calculation and can well keep the edge structure, while the texture background is smoothed. The pixel edge length is calculated as shown in the following formula:

(2) $$\begin{array}{c} L\left(z,l\right)=\left\{\begin{array}{cc} \text{max}\left(L\left(w,t\right)+1\right), & \text{if}\left|\left(w-z\right)\left(t-l\right)\right|<=1\text{ and }X\left(w,t\right)=X\left(z,l\right),\\ 0, & \text{for else}. \end{array}\right) \end{array}$$

where *L*(*w*, *t*) is the edge length of the pixel point (*w*, *t*), calculated by recursion. If the gray value of the pixel is the same as that of the neighboring pixels, the pixel edge length of the pixel is the largest edge length value of the neighboring pixels plus one.

The pixel edge length is introduced into the weight calculation formula. The weights are calculated as shown in the following formula:

(3) $$\begin{array}{c} m=\text{exp}\left[-\frac{{\left(x-z\right)}^{2}+{\left(y-l\right)}^{2}}{2\sigma_{d}^{2}}-\frac{{\left\|X\left(x,y\right)-X\left(z,l\right)\right\|}^{2}}{2\sigma_{r}^{2}}-\frac{\left|L\left(z,l\right)-L\left(x,y\right)\right|}{2\sigma_{l}^{2}}\right]. \end{array}$$

where *σ*_*l*_ is the value of the smoothing weight associated with the pixel edge length.

The improved bilateral filtering algorithm smooths the texture background, while the thin scratches on the wood panel surface are better maintained, as shown in Figure 2. In order to quantitatively evaluate the effect of texture smoothing of the improved bilateral filtering algorithm, the Structural Similarity (SSIM) index is used for evaluation, and the closer its value is to 1, the higher the similarity of the two images. As can be seen from Table 1, the improved bilateral filtering algorithm can maintain the defect characteristics better while smoothing the texture background.

## 4. Algorithm of This Paper

Faster R-CNN consists of four parts. The proposed improved Faster R-CNN model combines a variable convolutional residual network, ResNet50, with an improved path aggregation feature pyramid network (PA-FPN) and feeds the extracted multiscale feature maps into attention region proposal network (A-RPN) with a fused convolutional attention module. The extracted multiscale feature maps are entered into the A-RPN with ROI Align to further complete the detection of plate defects. The model structure is shown in Figure 3.

### 4.1. Multiscale Feature Extraction Network

The work in this paper detects defects in plate images. However, cut plate defects are characterized by large scale variations and different shapes. The existing Faster R-CNN directly utilizes the features output as the subsequent classification regression. As the feature information contained in the shallow layer network is easily lost, there will be small defects appearing as missed detections. Based on the FPN, PA-FPN is proposed to be combined with the variable convolutional residual network ResNet50 to improve the model's ability to represent the features of multiscale defects.

PA-FPN adds bottom-up path aggregation to the FPN to preserve shallow features considering the importance of shallow network information for small target detection. As shown in Figure 4, the solid arrows indicate the bottom-up feedforward computation of the FPN to generate features {*C*_2_, *C*_3_, *C*_4_, *C*_5_}. The solid arrows indicate the bottom-up computation of the FPN to generate features. FPN adds top-down computation to build a feature pyramid to acquire feature with rich semantic information {*U*_2_, *U*_3_, *U*_4_, *U*_5_}. The FPN adds top-down computation and lateral connectivity to build feature pyramids to obtain multiscale feature maps with rich semantic information. To preserve the shallow feature of the image, a bottom-up path aggregation is added, as shown by the dashed arrow in Figure 4, to better preserve the shallow feature information with less than ten layers of feature aggregation, and to obtain {*T*_2_, *T*_3_, *T*_4_, *T*_5_}. For subsequent classification and regression of the predicted targets, where *T*_2_ is the same as *U*_2_, PA-FPN will improve the adaptability of the model to detect defects at different scales in the image, especially to small-sized wood panel defects.

### 4.2. ResNet50 Network with Deformable Convolution

Faster R-CNN feature extraction layer generally adopts multilayer convolutional networks, and commonly used network structures include VGG-16, ResNet50, and ResNet101. ResNet network introduces short connections to addressing the challenges of gradient disappearance and gradient explosion while deepening the network to ensure the improvement of the overall network performance. Therefore, ResNet50 is used as the feature extraction layer in this paper.

To increase the robustness of detection to different shapes of wood panels, Deformable Convolutional Networks (DCNs) are introduced into ResNet50 in this paper. Deformable Convolution is to add displacement variables to the traditional convolutional layers. The feature map is combined with the displacement variable to form a new feature map, which changes the perceptual field from the original rectangular region to a polygonal region with variable shape, thus improving the network's ability to extract features from targets of different shapes. Displacement variables can be obtained by backpropagation learning. This can effectively cope with changes in geometry and improve the shape modeling capability of the convolutional neural network.

Raw convolutional layer output is shown as

(4) $$\begin{array}{c} j\left(u_{0}\right)=\sum_{u_{x}\in ℜ}m\left(u_{x}\right)\cdot i\left(u_{o}+u_{x}\right), \end{array}$$

where *u*_*o*_ is the coordinate of the pixel point at the center of the convolution kernel. ℜ is the image area covered by the convolution kernel. *u*_*x*_ are the coordinates of the pixel points within the convolution kernel other than *u*_*o*_.

Output of the convolution layer after introducing the offset is shown as

(5) $$\begin{array}{c} j\left(u_{0}\right)=\sum_{u_{x}\in ℛ}m\left(u_{x}\right)\cdot i\left(u_{o}+u_{x}+\Delta u_{x}\right). \end{array}$$

With the introduction of offsets, the grid points of the original convolution kernel can vary in the *i* and *j* directions. Therefore, the deformable convolution layer has a richer feature representation capability. Compared with the original convolution, the deformable convolution can approximate the real shape of the target object by positional transformation in the sampling point distribution, so the deformable convolution has stronger feature extraction ability.

ResNet50 consists of 5 phases. Each stage consists of 2 basic residual blocks. The role of the residual block1 is to change the dimensionality of the network, and the residual block2 is to deepen the network depth. By introducing deformable convolution into ResNet50, the 3 × 3 convolution layer in the residual block is replaced with a deformable convolution layer, and the result is shown in Figure 5.

After replacing the original convolution layer of Faster R-CNN with a shape-shifting convolution, ResNet50 can automatically adjust the scale or perceptual field. This engagement allows for better characterization of plate trace defects and improves the robustness of the network in detecting defects of different shapes.

### 4.3. RPN Networks with Converged Attention

#### 4.3.1. Anchor Settings

Regional recommendation network RPN is a significant improvement of Faster R-CNN, which assigns *k* anchor boxes to each point of its input feature map by sliding window, and further recommends target regions by classifier and bounding box regression principle. When setting the anchor, not only the scale parameter of different scales, but also the aspect ratio parameter of the target should be considered based on the base anchor box size.

To generate anchor frames that are closer to the actual target defect size in the dataset and to improve the performance for position regression, k-means provides guidance on the setting of anchor size. The clustering is performed for the target defect size in a specific dataset; that is, the intersection ratio (IOU) between the manually labeled ground-truth and the cluster center is calculated. The clustering is performed with the 1-IOU distance metric, and the RPN is guided to generate anchors that better match the shape of the actual defect to further localize and detect the defect. The implementation process is as follows.

(1) Given *w* clustering centroids (*M*_*x*_, *B*_*x*_), *x* ∈ {1,2,…, *w*}, where *M*_*x*_, *B*_*x*_ denote the width and height of anchor. Since their positions are not fixed, the coordinates (*i*, *j*) of the centroids are not given.
(2) The file containing the target locations generated during the dataset annotation process has (*i*_*y*_, *j*_*y*_, *m*_*y*_, *b*_*y*_),  *y* ∈ {1,2,…, *T*}. That is, the coordinates of the ground-truth are relative to the original map, where (*i*_*y*_, *j*_*y*_) are the coordinates of the centroid of the box. (*m*_*y*_, *b*_*y*_) is the width and height. *T* is the number of labeled boxes.
(3) Calculate the distance *d* between the labeled boxes in the dataset and the centroids of the *w* clusters.
  (6) $$\begin{array}{c} d=1-IOU\left[\left(i_{y},j_{y},m_{y},b_{y}\right),\left(i_{y},j_{y},M_{x},B_{x}\right)\right]. \end{array}$$
The labeled box is divided to its nearest (*M*_*x*_, *B*_*x*_) point according to the size of *d*.
(4) Until all labeled boxes are assigned, calculate the final cluster centroids for each cluster.
  (7) $$\begin{array}{c} M_{x}^{\prime }=\frac{1}{T_{x}}\sum m_{x},\;B_{x}=\frac{1}{T_{x}}\sum b_{x}. \end{array}$$
(5) Stop the iteration when (*M*_*x*_, *B*_*x*_) changes very less. For the plate defect dataset, a more suitable aspect ratio of anchor is found by k-means clustering, which is {0.25, 0.5, 1, 1.66, 2.1, 3.3}, respectively, to improve the stability of the prior frame generated by RPN. Experimentally, it is demonstrated that the increase in training time is not significant by increasing the number of anchors.

#### 4.3.2. A-RPN

In order to improve the model's focus on plate defect features and suppress features from complex backgrounds, A-RPN is used. The improved network can detect the location of defects more accurately under the complex background interference of plate images. As shown in Figure 6, after feature extraction, the results are fed into the A-RPN. Firstly, the feature *F* is obtained after 3 × 3 convolution of the input feature map. After that, the feature map is convolved along the convolutional block attention module (CBAM) to obtain finer features *F′′* for subsequent and more accurate target classification and regression by A-RPN.

CBAM consists of two complementary modules, which are connected to suppress features of complex backgrounds while highlighting defects and focus on the spatial location of defects in plate images against complex backgrounds. Channel attention focuses on the “what” of the target. By assigning more weight to channels containing more defect information and less weight to channels containing more background information, channel attention selects channels that contain useful defect features. Spatial attention tells the network “where” the defects are and helps the network locate the defects in the feature map. The proposed attention region recommendation network A-RPN can generate more accurate defect recommendation regions under the interference of complex backgrounds and further improve the target detection effectiveness of the model.

As shown in Figure 6, suppose that the input feature map is *F* ∈ *R*^*C*×*B*×*M*^, and the attention map is first obtained by the channel attention module *W*_*c*_ ∈ *R*^*C*×1×1^ . The *W*_*c*_ is weighted for each channel of the input feature *F*, and then the refined feature is obtained *F*′. Then, the attention map is obtained by the spatial attention module. *W*_*s*_ ∈ *R*^1×*B*×*M*^. *W*_*s*_(*F*′) and the features *F*′ are multiplied together to get *tF*^″^.

For the channel attention module, which focuses on “what is,” average pooling (represented by *U*_avg_ in the formula) and maximum pooling (represented by *U*_max_ in the formula) are carried out on the feature maps firstly, and two features are extracted to describe *F*_avg_^*c*^ and *F*_max_^*c*^. Secondly, these two different features are fed into the intermediate shared network layer separately. After the shared network is applied to the *F*_avg_^*c*^ and *F*_max_^*c*^ features, the corresponding elements of the two obtained features are summed, and then *W*_*c*_ ∈ *R*^*C*×1×1^ is acquired. The calculation formula is as follows:

(8) $$\begin{array}{c} W_{c}\left(F\right)=\sigma \left(U_{\text{MLP}}\left(U_{\text{avg}}\left(F\right)\right)+U_{\text{MLP}}\left(U_{\text{max}}\left(F\right)\right)\right)\\ =\sigma \left(M_{1}\left(M_{0}\left(F_{\text{avg}}^{c}\right)\right)+M_{1}\left(M_{0}\left(F_{\text{max}}^{c}\right)\right)\right). \end{array}$$

where the shared network layer represents a multilayer perceptron (MLP, denoted by *U*_MLP_ in formula.) containing two layers of the neural network. *σ* represents the sigmoid activation function. *M*_0_ and *M*_1_ represent the parameters of the two layers of the multilayer perceptron model. And *M*_0_ and *M*_1_ features between them are processed using ReLU as the activation function. Finally, *W*_*c*_(*F*) is multiplied with its input features to obtain the fine feature map adjusted by channel attention *F*′.

For spatial attention, the feature maps are obtained by average pooling and maximum pooling *F*_avg_^*s*^ ∈ *R*^1×*B*×*M*^ and *F*_max_^*s*^ ∈ *R*^1×*B*×*M*^, then the feature maps are merged, and the new spatial attention map is obtained using a 7 × 7 convolution kernel with a Sigmoid activation function *W*_*s*_(*F*).

(9) $$\begin{array}{c} W_{s}\left(F\right)=\sigma \left(g^{7\times 7}\left(\left[\left(U_{\text{avg}}\left(F\right)\right);U_{\text{max}}\left(F\right)\right]\right)\right)\\ =\sigma \left(g^{7\times 7}\left(\left[F_{\text{avg}}^{s};F_{\text{max}}^{s}\right]\right)\right). \end{array}$$

where *σ* represents the sigmoid activation function. *g*^7×7^ represents the convolution operation with a convolution kernel size of 7 × 7. Finally, *W*_*s*_(*F*′) is multiplied with its input features to obtain the final feature map *F*^″^.

### 4.4. Region of Interest Calibration (ROI Align)

In the original Faster R-CNN model using region of interest pooling (ROI Pooling) to roughly pool the candidate regions of different sizes into the same size feature map, this process generates quantization error twice. The steps are as follows:

1. Based on the input image, the candidate region is mapped back to the corresponding position of the feature map. The coordinates are rounded down to matrix coordinate values.
2. The obtained area is divided equally into *z* × *z* (7 × 7) cells (bins). The coordinates of the floating-point cells are quantized and rounded.

The impact of the deviations generated by the above two steps on the detection of small defects is huge. For example, the pixel size of surface defects for dirty spots is often 20 below. After feature extraction by the ResNet-50 pretrained network of deformable convolutional networks, both defects and images are scaled to 1/32 of the original image. A deviation of just 0.7 pixel can lead to a loss of information about this surface defect, also called the region mismatch (misalignment) problem.

In this paper, we use ROI Align to avoid region mismatch (misalignment) issue instead of rough ROI Pooling.

ROI Align differs from ROI Pooling not by simply quantifying and then pooling, but by using a regional feature aggregation approach to transform it into a continuous operation. This is shown in Figure 7.

1. Iterate over all candidate regions and keep the mapped candidate region floating point coordinates unquantized.
2. The candidate region is divided into *z* × *z* (2 × 2 in the figure) cells, and each cell is also not quantified.
3. Determine 4 positions of a sample point in each cell. The floating-point coordinates of the sampled points are calculated using a bilinear interpolation method to find the value of 4 positions. Then, the ROI output in a fixed dimension can be gotten.

where the large dashed grid represents the feature map (5 × 5). The solid grid is the variable-size ROI, that is, the candidate region. The 4 sampling points determined in each cell are obtained by dividing the cell into 4 small squares equally and taking the center points of the squares separately. With the above processing, the region mismatch problem can be avoided, and the model can obtain more accurate candidate feature regions. This can make the detection network further enhanced for fine defects detection and obtain higher accuracy.

## 5. Analysis of Experimental Results

### 5.1. Data Set

In this paper, LabelImg is used to calibrate the image samples. To improve the training effect and the generalization performance of the model, data enhancement methods are used for the dataset. Since changing different orientations and angles does not change the image sample features, this paper uses both horizontal flip and vertical flip2 data enhancement methods. In the annotation process, a total of 4956 target objects in 3216 images are annotated. All images are renamed according to VOC2007 data format and set to jpg format. Before training and testing, the images containing various types of defects (3216) were first normalized to 300 × 300 × 3 size (300 × 300 indicates the image resolution, and 3 means that there are 3 RGB color channels).

To generate the test dataset, 20% of the images from the annotated image dataset are selected as the test set. The test set contains all 5 types of defect images to be detected and approximately the same number of images for each defect type. The labeled images are fine-tuned, and the image information and xml format files are saved separately. The number of the surface defect images of the man-made board is shown in Table 2.

### 5.2. Experimental Platform and Model Parameters

This experiment is based on 64-bit windows 10 operating system: GPU model is 11 GB GPU Ge Force GTX 1080Ti. Memory is 32 GB DDR4. Hardware, and software platform is built by python language, using PyTorch based deep learning framework and using CUDA version 8.0 computing framework.

After the selection of the tuning parameters, some of the final model training parameters are as follows: the memory factor (momentum) is 0.9, and the small batch size is 16. The maximum number of iterations is 1000. And the learning rate is 0.0003. The number of decay steps is 400 and 800, and the weight decay factor is 0.0001. In the RPN network, a sufficient number of proposals generated will avoid the defect detection to a certain extent, but all of them will be used for subsequent training, which will slow down the training speed and increase the computational burden of training. Therefore, we need to use NMS to complete the proposal selection and set the threshold parameter of nonmaximum suppression for RPN network training to 0.7. The number of proposals after NMS is set to 2000.

### 5.3. Experimental Results

To verify the performance for detecting defects on real surfaces and its ability to generalize the defect detection to different texture backgrounds, the trained model is tested on a test set of plates with scratch defects. The results of scratch detection on the test set using the model proposed in this paper are shown in Table 3.

The number of missed detections in Table 3 refers to the number of images where scratches exist on the surface of the wood panel but are not recognized by the model. The number of false detections refers to the number of images where the model incorrectly identifies the grain background as scratches. The positive detection rate represents the percentage of images where the model correctly identifies the scratches on the wood panel surface to the total number of images. As can be seen from Table 3, the positive detection rate of the model proposed in this paper is 96.51% on the test set. Among them, when the texture background of the image to be detected is the same as that of the training set, the positive detection rate of real scratches reaches 98.5%, which fully verifies the effectiveness of the scratch generation method proposed in this paper as a data enhancement method. When the texture background is different from the training set, the positive detection rate decreases, indicating that the detection ability of the model decreases when the texture background changes. However, the positive detection rate is still around 91.6%, indicating that the proposed model provides a decent generalization ability in detecting scratches on wood panel surfaces with different texture backgrounds.

The experiments were conducted on the plate dataset as shown in Figure 8. As can be seen from the figure, the final AP value is 89.07% when the original Faster R-CNN is applied for multiscale defect detection. On top of that, the AP of Faster R-CNN + ResNet50 with deformable convolution is improved by 1.69%, while the AP value of ResNet50 with deformable convolution network combined with ROI Align is improved by 3.36%. Then, after incorporating the attention CBAM module into the model, the AP increased by 6.52% compared to the original model, reaching 95.59%. This indicates that using Attention CBAM focuses on defective features and suppresses features of complex backgrounds. In addition, using PA-FPN to extract multiscale features can better improve the detection results of multiscale defects, especially small target defects. Currently, the AP improves 9.31% over the original model to 98.38%. It is worth noting that the AP values of fusing channel attention and spatial attention into RPN based on the combination of RPN are 92.33% and 91.41%, respectively. This indicates that fusing only channel attention has little effect on the detection effect of the model, and fusing only spatial attention decreases the detection result of the model by 0.92%.

To verify the sensitivity of the key parameters of the model, ablation experiments are performed on the number of deformable convolution layers. The experimental results are shown in Table 4. In the different strategies, 3, 4, 5 indicates replacing the 3 × 3 convolution of ResNet50 stages 3–5 with the deformable convolution. From the experimental results, adding shape-shifting convolution layer in the case of unclear semantic information may lead to an increase in false positive samples, which results in lower accuracy and recall. Moreover, increasing the number of deformable convolutional layers will lead to an increase in computation, training time, and average detection time of a single image. Therefore, in this paper, only the 3 × 3 convolution in the stage 5 of ResNet50 is replaced with the deformable convolution to ensure that the displacement of the deformable convolution kernel can be learned from better features and reduce the model computation.

The trained model is used to test newly taken 197 plates with a processed size of 300 × 300 pixels, and the specific test results are shown in Figure 9. It can be seen that this paper can experiment plate defect detection with high detection accuracy.

To further validate the superiority of the proposed model for defect detection, comparative experiments are conducted for the existing defect detection methods.

As can be seen from Table 5, the recognition accuracy and recall rate of the proposed model are better than those of other algorithms, and compared with Cascade R-CNN, CBNet, and DetectoRS, which have better performance in two-stage target detection network, the proposed model has 3.15% higher accuracy and 2.02% higher recall rate compared with the best performance. This indicates that the improvements proposed in this paper have a large improvement on the model plate defect detection capability. The proposed model has improved training time and average detection time for a single image compared with U-Net, EfficientDet, and YOLOv4 using the lightweight backbone network VGG-16, but the accuracy and recall rate are much higher than them. In addition, the average inspection time of the proposed model is 0.4 s, which can meet the real-time requirements of wood panel processing production line.

## 6. Conclusion

An improved Faster R-CNN-based defect detection algorithm is proposed for identifying and locating surface defects for plates with complex textures. To enhance the model's ability to detect defects in different texture backgrounds, this paper proposes 4 improvements: (1) an improved bilateral filtering algorithm is proposed to smooth the image texture background. (2) A PA-FPN structure is used to fuse the multilayer features to obtain a multiscale feature map to express more complex semantic information, which is better for multiscale crack detection especially for small-scale defects. (3) RPN incorporates the attention module CBAM to improve the weight of the network for crack defects and indistinguishable samples, which improves the model's ability to distinguish defects from the background and improves the detection accuracy well. (4) The introduction of deformable convolution improves the feature extraction ability of the model for different scratch shapes.

The model proposed in this paper was tested on a real panel surface defect dataset, and the average positive detection rate of the model reached 95.71%, and the positive detection rate was 90% when tested using a new textured background wood panel image, showing that the model has good generalization capability. The comparison experiments proved that the improved model has a huge improvement in the detection ability of board defects. Comparing the model with other algorithms with superior performance verifies the superiority of the proposed model for the detection of panel defects. The next step will be to continue to investigate higher accuracy target detection algorithms and further explore how to enhance the defect features to suppress the interference of the background.

## Figures and Tables

**Figure 1:** Different plates.

**Figure 2:** Part of the surface texture of the veneer panel schematic.

**Figure 3:** Improved Faster R-CNN based surface defect detection algorithm for plates.

**Figure 4:** Block diagram of PA-FPN.

**Figure 5:** Residual block after introducing deformable convolution.

**Figure 6:** Regional recommendation network detection model with fused attention CBAM.

**Figure 7:** ROI Align principle.

**Figure 8:** Performance of plate image detection based on Faster-RCNN algorithm.

**Figure 9:** Detection results for multiple defects.

**Table 1:** Comparison of SSIM indicators with improved bilateral filtering algorithm.

Number of test images	Average SSIM value		Improvement (%)
	Bilateral filtering	Improved bilateral filtering	
200	0.8031	0.8862	10.35

**Table 2:** Number of partially defective images.

Defect type	Training set		Test set	
	Number of targets/image/images		Number of targets/image number of images	
Rough shavings	816	432	206	128
Watermark	776	526	201	146
Sand marks	803	569	293	132
Sundries	796	567	196	125
Gum spot	626	461	243	130

**Table 3:** Scratch defect detection results.

Defective texture background	Number of samples	Number of successful detections	Number of misses	Wrong number of checks	Positive inspection rate (%)
Same as the training set	100	98	—	1	98.50
Unlike the training set	40	36	3	1	91.60
Total	140	134	4	2	96.51

**Table 4:** Effect of the number of deformable convolution layers on model performance.

Ablation experiments	Different strategies	Accuracy (%)	Recall rate (%)	Training time (h)	Average detection (s)
Number of deformable convolutional layers	3, 4, 5	92.16	85.38	22	0.61
	4, 5	96.64	89.23	18	0.52
	5 (√)	98.43	92.86	16	0.40

**Table 5:** Comparison of the model proposed in this paper with other algorithms.

Algorithm	Accuracy (%)	Recall rate (%)	Training time (h)	Average inspection time/image (s)
Classification network + attention U-Net	85.27	83.36	6	0.32
Mask R-CNN	94.55	89.23	11	0.35
Cascade R-CNN	92.16	86.70	18	0.52
CBNet	94.50	89.58	19	0.57
DetectoRs	95.28	90.84	16	0.43
EfficientDet	89.74	85.41	8	0.23
YOLOv4	87.67	84.35	5	0.11
The model proposed in this paper	98.43	92.86	16	0.4

## Data Availability

The labeled datasets used to support the findings of this study are available from the corresponding author upon request.
